RETRACTED

# Study on the Effects of Orthodontics on Anterior Tooth Displacement in Patients

**DOI:** 10.1155/2022/6544895

**Published:** 2022-06-10

**Authors:** Beibei Zhang, Minqiu Cai, Fangchao Ruan, Zigen Chen

**Affiliations:** ^1^Department of Stomatology, The First People's Hospital of Wenling, Wenling 317500, Zhejiang, China; ^2^Department of Stomatology, Taizhou Enze Medical Center Luqiao Hospital, Taizhou 318050, Zhejiang, China

## Abstract

**Objective:**

The purpose of this study was to investigate the therapeutic effect of orthodontic treatment on anterior tooth displacement caused by periodontal disease.

**Methods:**

A prospective study was performed in 86 patients with anterior tooth displacement caused by periodontal disease. These patients were divided into the experimental group and the control group according to the intervention methods. For the control group, patients were treated with conventional therapy. The experimental group used straight wire orthodontic technique for orthodontic treatment on the basis of conventional treatment. Comparisons were performed between two groups in term of bleeding index, alveolar bone height, anterior tooth coverage, periodontal pocket depth, probing depth, clinical crown length, tooth root length, inflammatory cytokines levels, and orthodontic satisfaction.

**Results:**

Comparison of bleeding index, alveolar bone height, anterior tooth coverage, periodontal pocket depth, probing depth, clinical crown length, tooth root length, and inflammatory cytokines levels between two groups before treatment indicated that there were no statistical differences (all *P* > 0.05). After treatment, bleeding index, alveolar bone height, anterior tooth coverage, periodontal pocket depth, probing depth, clinical crown length, and serum levels of IL-6 and TNF-*α* in the experimental group were lower than those in the control group (all *P* < 0.05), while the serum level of IL-2 in the experimental group was more than that in the control group (*P* < 0.05). Also, there was no difference for tooth root length between two groups. Moreover, compared with the control group, orthodontic satisfaction in the experimental group was significantly increased.

**Conclusion:**

The efficacy of orthodontic treatment in patients with anterior tooth displacement caused by periodontal disease is higher than that of only using conventional therapy, as it helps improve their periodontal health, alveolar bone height, clinical crown length, inflammatory factor levels, and orthodontic satisfaction of patients.

## 1. Introduction

Periodontal disease is a common oral disease. More than 90% of the general population is reported to have periodontal disease, the incidence of which increases with age, and it is caused by bacterial infection in the oral cavity that leads to destruction of periodontal tissue, which in turn leads to fragmentation and displacement of anterior teeth, as well as enlarged gaps and other symptoms [1, 2]. Studies have shown that patients with periodontal disease may have pathologic tooth displacement, such as anterior tooth displacement [3]. Anterior tooth displacement not only affects the normal chewing function of patients but also affects facial aesthetics. Some patients with severe symptoms may even experience tooth loss.

RETRACTED

Currently, the main treatment options for anterior tooth displacement due to periodontal disease include conventional periodontal therapy, medication, periodontal tissue regeneration, and surgery. Previous studies have shown that it is difficult to achieve the desired clinical outcome using conventional treatment [4]. Orthodontic treatment is used clinically in patients with anterior tooth displacement. Orthodontic treatment has been reported to enhance the appearance and function of teeth by moving or straightening these pathological teeth [5, 6]. However, few studies have shown the effect of orthodontic treatment on anterior tooth displacement after periodontal disease. In this context, the aim of this study was to investigate the effect of orthodontic treatment on patients with anterior tooth displacement after periodontal disease. The study experiment divided the patients into experimental and control groups according to the intervention method. The control group was treated conventionally. The experimental group underwent orthodontic treatment on the basis of conventional treatment. The orthodontic satisfaction was significantly higher in the experimental group compared to the control group. The results of this study will provide a basis for the clinical treatment of anterior tooth displacement caused by periodontal disease [7–10].

## 2. Materials and Methods

### 2.1. General Information

This study was conducted on 86 patients diagnosed with anterior tooth displacement caused by periodontal disease in the Department of Stomatology, The First People's Hospital of Wenling from January 2017 to June 2020. This was a retrospective study. These patients were divided into the experimental group and the control group. There were 43 patients in each group. The conventional periodontal treatment was performed in both groups [11]. Moreover, patients from the experiment group received the orthodontic treatment. All patients included in this study signed the informed consent. This trial was approved by the Ethics Committee of The First People's Hospital of Wenling [12–15].

RETRACTED

Inclusive criteria are as follows: anterior tooth displacement caused by periodontal disease was diagnosed according to the Diagnostic Criteria of Guidelines for Prevention and Treatment of Periodontal Disease in China. Patients were accompanied by tooth displacement, elongation of anterior teeth, masticatory dysfunction, obvious protrusion of anterior tooth, deep overbite, atrophy of periodontal tissue, and other symptoms. The age was between 18 and 60 years old. Patients never received orthodontic treatment before. Patients were able to effectively cooperate with this treatment.

Exclusive criteria are as follows: severe liver and kidney dysfunction, or cardiovascular and cerebrovascular diseases were found; patients had contraindications of orthognathic surgery. Patients took antibiotics and immunosuppressive drugs for a long time. Patients had allergic reactions to the drugs in this study. Anterior tooth displacement was caused by other reasons besides periodontal disease. One or more teeth were missing per quadrant. Patients were with incompleted information. Patients were pregnant and breastfeeding [16–19].

### 2.2. Treatment Methods

The details of conventional periodontal treatment are as follows: patients received oral cleaning including effective oral cleaning methods and hygiene-related knowledge and education. Patients also underwent periodontal and root surface treatment, which consisted of supragingival cleansing, subgingival scraping, caries removal and bad restoration, periodontal pocket washing, tooth root surface grinding, and restoration of periodontal- and endodontic-affected tissues. Moreover, antibiotics were performed in patients if necessary [20, 21]. Besides the conventional periodontal treatment, patients in the experiment group underwent orthodontic treatment. The details are as follows: the straight wire orthodontic technique is used to correct the patient's teeth. The bracket should be bonded to the incisor teeth as close as possible without the ring; nickel-titanium round wire was used to adjust the uniformity of the patient's teeth. The multicurved labial arches pressed down the upper and lower dental cusps of patients and the teeth were ligated continuously to enhance the stability. The anterior teeth were adducted with a rubber chain. Finally, the orthodontic force was appropriately adjusted during the process of treatment [22].

### 2.3. Outcome Measures

Before and after treatment, it was compared between the control group and experimental group in terms of bleeding index, alveolar bone height, anterior tooth coverage, periodontal pocket depth, probing depth, clinical crown length, and tooth root length [23–26].

RETRACTED

Serum levels of IL-2, IL-6, and TNF-*α* were detected using the enzyme-linked immunosorbent assay (ELISA). The operating steps were strictly conducted following the instructions in assay kits. IL-2, IL-6, and TNF-*α* levels were compared between two groups.

The orthodontic satisfaction of patients was evaluated according to the report by Shen et al. [7]. The items consisted of speech function, chewing function, retention function, and aesthetic comfort. The total scores were 100 points. Less than 60 scores suggested unsatisfactory. Scores between 60 and 90 suggested general satisfaction. More than 90 scores suggested very satisfied. Total satisfaction = basic satisfaction + very satisfaction.

### 2.4. Statistical Analysis

All data were analyzed using the SPSS statistical software version 23.0. The enumeration data were calculated as number/percentage (n/%). The comparison was exploited using the chi-square test. The measurement data were expressed as mean ± standard deviation. *T*-test was exploited for the intergroup comparison. The difference was statistically significant when the *P* value was less than 0.05.

## 3. Results

As shown in Table 1, there were no differences regarding gender, age, course of disease, underlying disease, index of bleeding, degree of deep overbite, and anterior teeth displacement between the two groups (all *P* > 0.05).

As shown in Tables 2–4, before treatment, there were no statistical differences between two groups in term of bleeding index, alveolar bone height, anterior tooth coverage, periodontal pocket depth, probing depth, clinical crown length, tooth root length, and inflammatory cytokines levels. After treatment, there were obviously statistical differences between the two groups regarding the bleeding index, alveolar bone height, anterior tooth coverage, periodontal pocket depth, probing depth, clinical crown length, and inflammatory cytokines levels (all *P* < 0.05). No difference was found in tooth root length between the two groups. In addition, the orthodontic satisfaction of patients in the experimental group was significantly higher than that in the control group.

Also, there was a significant difference between the two groups (*P* < 0.05), as seen in Table 5.

## 4. Discussion

With the enhancement of people's consciousness of oral health, more and more persons are conscious of the harmful effects of periodontal disease, which has a serious impact on the oral health of people. The measures are required to be performed to improve the oral health and teeth of patients. Anterior teeth displacement caused by periodontal disease was one of the most common conditions of the oral cavity. Some studies reported that patients with anterior teeth displacement after periodontal disease could benefit from the orthodontic treatment. However, not enough evidence was provided to confirm this opinion. In recent years, orthodontic treatment was performed for these patients with anterior teeth displacement caused by periodontal disease in our hospital and a lot of experiences were accumulated. In this study, the effects of orthodontic treatment on anterior tooth displacement in patients with periodontal disease were investigated. The results showed orthodontic treatment combined with conventional therapy achieved better effects in the bleeding index, alveolar bone height, anterior tooth coverage, periodontal pocket depth, probing depth, and clinical crown length than conventional treatment alone, suggesting orthodontic treatment was more effective, so it helped improve the periodontal health. Lee et al. reported that the indices regarding periodontal tissue of the affected tooth in the observation group were better than they were in the control group after treatment, which was highly in accordance with the results of this study.

RETRACTED

Many studies showed that the excessive accumulation of bacteria could further lead to the transformation of subgingival plaque into more aggressive pathogen populations, resulting in more severe periodontitis. The main therapeutic methods included the elimination of inflammation, control of disease development, and stabilization of the local microenvironment in the periodontal tissue. Inflammatory cytokines play an important role in regulating chronic inflammation responses. It was reported that the expression levels of IL-2, IL-6, and TNF-*α* were associated with the severity in patients with anterior teeth displacement caused by periodontal disease. IL-2 is a kind of cell growth factor in the system of immune. It was shown that the increased level of IL-2 suggested an increase in the immunity of the body. IL-6 is another inflammatory cytokine. It could act on vascular endothelial cells and regulate the inflammatory response. It was observed that the increased level of IL-6 suggested that there was a state of pathological damage in the body. TNF-*α* is considered a killing mechanism for cell death in cancers. It not only has anti-infection but also has antitumor effects. It was found that the increased level of TNF-*α* suggested an inflammatory state. In this study, compared with the IL-2 level was significantly higher and the IL-6 and TNF-*α* levels were lower in the experimental group after therapy, indicating that the levels of inflammatory cytokines were improved, and the immunity was enhanced after orthodontic treatment plus conventional treatment.

RETRACTED

There were some limitations in this study. First, this study had short-term results, and no further long-term outcome measurement was collected. Future studies are required to elaborate on the follow-up data. Second, the sample size was relatively small, and it may influence the findings. Third, this was a single-centre study. All the data were collected from The First People's Hospital of Wenling. Also, it may influence its generalization to other hospitals. Finally, it failed to conduct multicenter randomized controlled clinical trials with a large sample, as a result of a retrospective study.

In conclusion, by performing this study, it has been proved that orthodontic treatment combined with conventional treatment could significantly improve anterior teeth displacement caused by periodontal disease showing higher efficacy and satisfaction than conventional treatment alone. However, these conclusions were still required to be confirmed by more high-quality studies.

## Figures and Tables

**Table 1:** Comparison of basic data between two groups.

Parameters	Experimental group (*N* = 43)	Control group (*N* = 43)
Male/female (n)	27/16	24/19
Age (years)	48.5 ± 5.6	49.3 ± 6.1
Hypertension (n)	9	7
Diabetes (n)	8	11
Course of disease (years)	6.1 ± 1.4	5.8 ± 1.1
Anterior teeth displacement (n)		
Teeth twist	12	14
Lip forward	15	19
Anterior teeth elongation	16	18
Titled teeth	25	22
Index of bleeding (n)		
0–3 grade	21	23
4–5 grade	22	20
Degree of deep overbite (n)		
I	23	20
II	13	15
III	7	8

**Table 2:** Comparison of the periodontal index and anterior alveolar bone height between two groups.

Groups		Bleeding index (%)	Anterior tooth coverage (mm)	Alveolar bone height (mm)	Periodontal pocket depth (mm)
Experimental group	Before treatment	89.4 ± 7.1	6.8 ± 1.7	5.7 ± 0.8	5.8 ± 0.9
	After treatment	23.2 ± 3.8	2.1 ± 0.6	2.7 ± 0.4	2.3 ± 0.5
Control group	Before treatment	88.7 ± 6.4	6.6 ± 1.4	5.9 ± 0.7	5.6 ± 0.6
	After treatment	36.5 ± 4.6	3.6 ± 0.8	3.7 ± 0.6	3.5 ± 0.7

**Table 3:** Comparison of probing depth, clinical crown length, and tooth root length between two groups.

Groups		Probing depth (mm)	Clinical crown length (mm)	Tooth root length (mm)
Experimental group	Before treatment	3.3 ± 0.6	8.8 ± 1.9	11.5 ± 1.3
	After treatment	2.0 ± 0.3	2.1 ± 0.6	11.1 ± 1.2
Control group	Before treatment	3.6 ± 0.5	8.7 ± 1.7	11.6 ± 1.1
	After treatment	2.7 ± 0.6	8.1 ± 1.2	11.3 ± 1.0

**Table 4:** Comparison of Inflammatory cytokines levels between two groups.

Groups		IL-6 (pg/mL)	IL-2 (ng/mL)	TNF-*α* (ng/mL)
Experimental group	Before treatment	203.5 ± 40.2	1.8 ± 0.7	3.9 ± 0.8
	After treatment	149.3 ± 30.5	4.2 ± 1.0	1.4 ± 0.3
Control group	Before treatment	197.4 ± 38.6	2.1 ± 0.8	3.8 ± 0.7
	After treatment	174.9 ± 32.7	3.0 ± 0.9	2.7 ± 0.5

RETRACTED

**Table 5:** Comparison of orthodontic satisfaction of patients between two groups (n (%)).

Groups	Very satisfied	Generally satisfied	Unsatisfactory	Total satisfaction rate
Experimental group (*N* = 43)	31 (72.1)	10 (23.3)	2 (4.7)	41 (95.3)
Control group (*N* = 43)	12 (27.9)	17 (39.5)	14 (32.6)	29 ( 67.4)

## Data Availability

The experimental data used to support the findings of this study are available from the corresponding author upon request.
